This article has been retracted.

# Clinico-histopathologic and outcome features of cutaneous infundibular keratinizing acanthoma: a case report and literature review

**DOI:** 10.1186/1477-7819-12-173

**Published:** 2014-06-03

**Authors:** Abbas Tavasoly, Hossein Gholami, Amir Rostami, Ali Anissian, Seyed Rashid Touni, Pooyan Khaleghian, Aram Mokarizadeh, Javad Javanbakht, Alireza Nasoori

**Affiliations:** 1 Department of Pathology, Faculty of Veterinary Medicine, Tehran University, Tehran, Iran; 2 Department of Clinical Science, Faculty of Veterinary Medicine, Tehran University, Tehran, Iran; 3 Department of Veterinary, College of Agriculture, Abhar Branch, Islamic Azad University, Abhar, Iran; 4 Faculty of Veterinary Medicine, Urmia University, Urmia, Iran; 5 Graduated of Faculty of Veterinary Medicine, Garmsar Branch, Islamic Azad University, Garmsar, Iran; 6 Department of Immunology, Faculty of Medicine, Kurdistan University of Medical Sciences, Sanandaj, Iran; 7 Graduate of Veterinary Medicine, Faculty of Veterinary Medicine, Karaj Branch, Islamic Azad University, Rajaee shahr, Moazen Boulevard, Karaj, Alborz, Iran; 8 Department of Pathobiology, Faculty of Veterinary Medicine, Tehran University, Tehran, Iran

**Keywords:** IKA, Keratin, Dog, Histopathology, Tumor

## Abstract

The infundibular keratinizing acanthoma (IKA) is a rare epithelial benign keratin-containing neoplasm of hair follicles. The purpose of this study was to evaluate the defining histopathologic architecture of IKA. A typical IKA consisted of a keratin-filled crypt in the dermis and subcutis that opened to the skin surface. Most of this tumor occurred on the back, neck, head, and the shoulders. Microscopically, the dermal nodules were focally contiguous in both the dermis and subcutis. Furthermore, most histological lesions are consistent with a simple or multiloculated cyst filled with keratin and lined by a wall of stratified squamous epithelium; keratin appears as a concentric lamellar mass, with a keratotic pearly aspect. Histological examination of the cutaneous lesions revealed that the growths were comprised of IKA. IKA of man and dog were compared, and it was concluded that although they are similar in many respects, they are not identical entities. To the best of our knowledge, this is the first report on the prevalence of IKAs among the population of owned dogs in Iran.

## Background

The cutis is continuously exposed to a wide variety of chemical and physical insults and other environmental factors and, therefore, is prone to neoplastic proliferation. In canines, approximately 30% of all neoplasms are reported to arise in the skin [1,2]. Neoplasm is the most common disease of companion animals, reaching 15 to 30% in dogs and 26% in cats, and eventually leads to death or euthanasia [3].

Acanthoma is a squamous cell tumor that may be malignant but well-differentiated, benign, or non-neoplastic. In humans, it occurs more frequently in a combined form which is called keratoacanthoma and adenoacanthoma. In the dog, two types of tumors with an acanthoma component have been described: infundibular keratinizing acanthoma (IKA), which is a common cutaneous tumor similar to keratoacanthoma, and melanocytoma acanthoma, a rare type of tumor described only once in the veterinary literature [4].

The IKA (synonyms are: intracutaneous cornifying epithelioma, keratinizing epithelioma, keratoacanthoma) arises from the upper part of the hair follicle so it may have a pore opening onto the surface. IKA is a rare epithelial benign follicular canine neoplasm that evolves rapidly, forming a solitary or multiple firm, flask-shaped cystic nodules with keratin in their centers [5,6].

In the IKA, the neoplastic growth into the surrounding dermis is by blunt cords of well-differentiated squamous epithelium with a continuous border of basal cells [7]. IKAs are benign follicular canine tumors that evolve rapidly, forming a solitary mass, or multiple firm, flask-shaped nodules with a central horn-filled cyst, that grow into the surrounding dermis through blunt cords of well-differentiated squamous epithelium surrounded by a continuous border of basal cells. In both neoplastic conditions, a frequent morphological finding is the occurrence of ‘horn pearls’ [8,9]. The aim of this study was to evaluate the defining histopathologic architecture of the IKA.

## Case presentation

A 4-month-old intact female brown splash Boston terrier was presented to the Small Animal Clinic of Tehran University. Dermatological examination revealed solitary, multiple and flask-shaped 1- to 3-cm-diameter nodules which were painful, firm, of unknown duration and of different sizes, with a central pore filled with keratin. The masses were located in the intradermal layer of the dorsal trunk, back, neck, head, shoulder and thorax, were dome-shaped, had an irregular surface, and were freely movable. No other clinical signs or evidence of metastasis were noted. The masses were excised completely under local anesthesia with minimal bleeding and the incision was closed using Vicryl 5.0 sutures. Post-operative recovery was uneventful. The biopsy consisted of masses of pale, greyish tissue with an irregular surface measuring 1 to 3 cm in diameter. Subsequent excisional biopsy samples fixed in 10% neutral buffered formalin and embedded in paraffin, and 4-μm-thick sections were stained with H&E and were pathologically evaluated at our institution.Microscopically, the dermal nodules were focally contiguous in both the dermis and subcutis. Most histological lesions are consistent with a simple or multiloculated cyst filled with keratin and lined by a wall of stratified squamous epithelium; keratin appears as a concentric lamellar mass, with a keratotic pearly aspect. Some spinous cells are arranged as epithelial cords or islands in the keratin mass (Figure 1A-D). Furthermore, the neoplastic growth into the surrounding dermis is by blunt cords of well- differentiated squamous epithelium with a continuous border of basal cells. The basal layer of the epithelial tumor nests showed cordlike expansion into the surrounding compressed dermis but without invasion of tumor cells across the basal lamina. Also, multifocal cords form variably-sized cysts lined by gradually keratinizing epithelium and are filled with lamellated keratin (horn cysts). In some regions, the proliferating cells were regularly restricted to the outermost one or two layers of tumor lobules while the keratinized central cells were devoid of proliferating cells (Figure 1A-D). A diagnosis of IKA was made. No recurrence of disease was noted during a follow-up period of eight months.

**Figure 1:** **Photomicrograph of the cutaneous infundibular keratinizing acanthoma.** Brown splash boston terrier dog. **(A-D)** Neoplasm consist of nests of well-differentiated squamous epithelium and nests of squamous epithelium with a continuous border of basal cells and also lesions are consistent with a simple or multiloculated cyst filled with keratin and lined by a wall of stratified squamous epithelium and keratin appears as a concentric lamellar mass, with a keratotic pearl aspect. H&E, 400×, Bar = 10 μm.

## Discussion

IKAs are uncommon benign follicular tumors in the dog. They can occur in young and middle-aged dogs with males being affected more than females. Clinical and histopathologic features of canine IKAs have not been recently described in the literature. Major textbooks of dermatopathology mention IKA only briefly. To our knowledge, only one prior study on IKA correlated histopathologic findings with biologic behavior. In that study, the authors focused on the histopathologic findings in the initial biopsies of lesions that resembled IKA versus those that did not (‘squamous cell carcinoma’). The majority of IKA lesions were left untreated and followed up to complete clinical resolution without additional histopathologic evaluation [4-6,8]. Furthermore, in according previously studies demonstrated that histopathology of skin has been documented to be useful in the diagnosis of several skin lesions [10-13].

Result from the proliferation of IKA neoplastic cells with a marked perifollicular orientation with the epithelial neoplastic component seen in the present tumor. The epithelial component of the tumor described here is a well-differentiated squamous epithelial growth with a distribution pattern of cytokeratins similar to those described in the normal epidermis and epidermis-derived tumors of humans, dogs, and cats [14,15]. This cytokeratin pattern is not inconsistent with hair follicles and/or follicular neoplasms [14]. Some of the lesions in the multiple IKA may have only a small cup-shaped depression or a dilated follicle filled with keratin with limited proliferation of squamous epithelium [16]. Occasionally, such features are seen in solitary lesions. It appears that involution occurs at an early stage in their development, so our findings were shown in parallel with the above results. Also, by the presence of the follicular, horn and epidermal cysts, our findings revealed relatively different frequencies compared to those reported in earlier investigations [17,18]. Moreover, our study demonstrated that the IKA of canines that are prevalent in other parts of the world are also prevalent in dogs in Iran. Our observation on the age of the dog affected by IKA and anatomical locations shows that there is no significant variation in these important parameters among Iranian dogs and dogs from other geographical areas.

The limitations of this study are the low number of cases, the fact that it was retrospective, and the lack of a gold standard for histologic diagnosis of IKA.

Because this tumor occurred in only one dog and there is little clinical data in the previous report, no conclusions concerning age, breed, sex, or site predilections can be made. The dog was in good health four months after tumor excision, and there was no evidence of local regrowth or metastasis. There appear to be no clinically distinctive features of canine IKA. The diagnosis of this neoplasm can be based on the histologic appearance of the tumor. Furthermore, this result would serve as an important reference in future investigations.

## Conclusions

In conclusion, this study described histopathology features of canine cutaneous IKA. We anticipate that the result of our study would be useful for veterinary practitioners and veterinary students across the nation. To the best of our knowledge, this is the first report on the prevalence of IKAs among the population of owned dogs in the Iran, contributing to the understanding of the histopathology and the risk factors associated with some dog tumors.

## Consent

Written informed consent was obtained from the owner of the patient for the publication of this case presentation and any accompanying images. A copy of the written consent is available for review by the Editor-in-Chief of this journal.

## Abbreviations

H&E: hematoxylin and eosin; IKA: infundibular keratinizing acanthoma.

## Competing interests

The authors declare that they have no competing interests.

## Authors’ contributions

AT and HGH participated in the histopathologic evaluation, performed the literature review, acquired photomicrographs, drafted the manuscript and gave the final histopathologic diagnosis. AR, AA, PKH, AM and AN designed and carried out all the experiments and were the principal investigators of the laboratory in which the research were performed and contributed to the interpretation of the data, edited the manuscript and made required changes. JJ performed sequencing alignment and manuscript writing. All authors read and approved the final manuscript.
